# Baicalin Ameliorates DSS-Induced Colitis by Protecting Goblet Cells through Activating NLRP6 Inflammasomes

**DOI:** 10.1155/2022/2818136

**Published:** 2022-08-16

**Authors:** Yanan Li, Jingyi Hu, Cheng Cheng, Feng Xu, Ryan Au, Lei Zhu, Hong Shen

**Affiliations:** Affiliated Hospital of Nanjing University of Chinese Medicine (Jiangsu Province Hospital of Chinese Medicine), Nanjing 210029, China

## Abstract

**Objective:**

Baicalin is an active compound found in many natural herbs and has been used to treat intestinal disorders such as diarrhea and colon cancer. In this study, we used a dextran sodium sulfate (DSS)-induced colitis mouse model to investigate baicalin's mechanisms in the treatment of colitis.

**Methods:**

3% DSS was administered through the drinking supply for 7 days to induce colitis followed by the administration of 5-aminosalicylic acid and baicalin at three different doses (25, 50, and 100 mg/kg, W/W) for an additional 7 days. Body weight, stool consistency, and colon length were recorded. Colon tissue was stained with hematoxylin and eosin (H&E) to be used for histopathological scoring. Cytokine levels of the colon tissue and serum were evaluated using real-time quantitative reverse transcription-polymerase chain reaction (qRT-PCR) and enzyme-linked immunosorbent assay (ELISA), respectively. mRNA expression and protein levels of tight junctions (TJs) were detected with qRT-PCR and Western blotting. Goblet cells and the mucosal layer of the colon were visualized by Alcian Blue/periodic acid-Schiff (AB/PAS) staining. Mucin 2 (MUC2) was evaluated in both mRNA expression and protein levels. Nod-like receptor pyrin domain-containing protein 6 (NLRP6) inflammasomes were detected by immunohistochemistry and Western blotting.

**Results:**

Treatment with baicalin significantly relieved colitis as evidenced by reversing both weight loss and colon length shortening. In addition, baicalin inhibited inflammation by reducing proinflammatory cytokines and protected the intestinal barrier by upregulating tight junction proteins. Moreover, goblet cell count and intestinal mucosa thickness were both significantly increased after baicalin treatment. Giving baicalin could upregulate the expression of NLRP6 and interleukin (IL-18) both in mRNA and protein.

**Conclusion:**

Baicalin ameliorates DSS-induced colitis by protecting goblet cells through activating NLRP6 inflammasomes.

## 1. Introduction

Ulcerative colitis (UC), first reported in 1895, is one of the two main types of inflammatory bowel disease (IBD) [1], and it is characterized by the presence of mucosal and submucosal inflammation limited to the colon and rectum [2]. Patients with UC often suffer from symptoms such as abdominal pain and bloody diarrhea. In the colon, the mucosal barrier is the first line of defense against attacks within the lumen. Previous studies have shown that the first step of UC development is dysfunction of the mucosal barrier [3]. Patients with subclinical UC often show a decreased number of goblet cells and a thinner mucosal barrier compared with healthy people [4]. Currently, many UC medications inhibit inflammation by rebalancing the immune system as opposed to targeting the mucosal barrier. As the goal of UC treatment shifts towards mucosal healing [5, 6], rebuilding the mucosal barrier is essential for intestinal barrier protection.

NLRP6 belongs to the nucleotide-binding oligomerization domain- (NOD-) like receptor (NLR) family of proteins [7]. Previous studies have shown that NLRP6 plays a vital role in intestinal homeostasis, which includes maintaining mucosal barrier function through regulating goblet cell mucus secretion [8] and regulating the gut microbiome through activating interleukin (IL)-18 [9]. Previous studies have also shown that dextran sodium sulfate (DSS)-induced colitis mice often show a decreased number of intestinal goblet cells and an absence of intestinal mucosa as a result of the inactivation of NLRP6 [10]. In addition, NLRP6-deficient mice are more susceptible to chemically induced colitis due to a compromised mucosal barrier. Because NLRP6 is central to regulating the mucosal barrier, targeting it may be a new strategy for UC treatment.

Previously, our research team found that Qingchang Huashi Formula, an herbal medication with many components, had a protective effect on goblet cells by promoting mucus secretion. This was especially apparent in Huang-Qin (*Scutellaria baicalensis Georgi*), which is an ingredient in Qingchang Huashi Formula [11]. In animal studies, many active components derived from Huang-Qin have been reported to be effective in the treatment of UC [12–15]. Of these active components, baicalin has been heavily researched and can be a potential candidate for new drug development. Many research groups have reported that baicalin could protect against chemically induced colitis in rats and/or mice through regulating the gut microbiota and immune system. Previously, we have shown that baicalin could rebuild the intestinal barrier by inhibiting the activation of the phosphatidylinositol 3-kinase (PI3K)/protein kinase B (AKT) pathway, ultimately upregulating the production of tight junction proteins, and downregulating the secretion of pro-inflammatory cytokines [16]. Also, we have found that baicalin may have prebiotic properties by promoting the growth of short-chain fatty acid (SCFA)-producing microbes, such as *Butyricimonas* spp., *Roseburia* spp., and *Subdoligranulum* spp. These microbes increase the levels of SCFAs in the colonic lumen to regulate the balance of regulatory T(Treg) and T helper 17(Th17) cells [17]. Although much research has been done on baicalin, its effects on mucosal function are still relatively unknown.

In order to research this topic further, we investigated the mechanisms of baicalin leading to the protective effects of the mucosal barrier. We found that baicalin not only prevented a decrease in the number of goblet cells but also maintained their function. Furthermore, we discovered that baicalin promotes the production of goblet cells in the mucosa by activating the NLRP6/IL-18 pathway. Thus, our findings provide a novel insight into the use of baicalin in the treatment of UC.

## 2. Materials and Methods

### 2.1. Reagents and Instruments

The following reagents and instruments were used in this study: dextran sodium sulfate (DSS; MW: 36000–50000; Cat. No. 160110; MP Biomedicals; Santa Ana, CA, USA), baicalin (Cat. No. B20570; Yuanye Bio-Technology Co., Ltd.; Shanghai, China), 5-aminosalicylic acid (5-ASA; Cat. No. A3537-25G; Sigma-Aldrich; St. Louis, MO, USA), anti-NLRP6 and anti-claudin-5 antibodies (Cat. No. ABF29, ABT45; Sigma-Aldrich; St. Louis, MO, USA), anti-caspase-1 and anti-ZO-1 antibodies (Cat. No. sc-56036, sc-33725; Santa Cruz Biotechnology, Inc.; Dallas, TX, USA), anti-MUC2 and anti-claudin-4 antibodies (Cat. No. ab272692, ab15104; Abcam; Cambridge, United Kingdom), anti-GAPDH antibodies (Cat. No. 60004-1; Proteintech Group Inc., Rosemont, IL, USA), HRP-labeled goat anti-rabbit IgG and HRP-labeled goat anti-mouse IgG (Cat. No. GB23303, GB23301; Servicebio Technology Co., Ltd.; Wuhan, China), TRIzol™ Reagent RNA Extractor (Cat. No. 15596018; Invitrogen; Waltham, MA, USA), HiScript II RT SuperMix for qPCR and ChamQ SYBR qPCR Master Mix (Cat. No. R323-01, Q311-02; Vazyme Biotech Co., Ltd.; Nanjing, China), PCR primers (Control No. QP-D09-01; Shanghai Jierui Bioengineering Co., Ltd.; Shanghai, China), and ELISA kit (Cat. No. EK206/3, EK201B, EK282HS; Multisciences (Lianke) Biotech Co., Ltd.; Hangzhou, China).

### 2.2. Animals

Forty-eight male C57BL/6J mice (18–22 g, 6–8 weeks old) were purchased from Zhejiang Vital River Laboratory Animal Technology Co., Ltd. They were housed in the Experimental Animal Center of Jiangsu Provincial Hospital of Traditional Chinese Medicine with a constant temperature of 24 ± 1°C, a constant humidity level of 55%–65%, and a 12-hour light/dark cycle. Mice were acclimated for seven days under normal environmental conditions, where their dietary intake, activity, posture, fur quality, and other health markers were observed. Unhealthy mice were excluded from this experiment. All experimental procedures were carried out in strict accordance with the “Guidelines for the Treatment of Experimental Animals.” This experiment has been approved by the Animal Ethics Committee of the Affiliated Hospital of Nanjing University of Chinese Medicine (Approval No. 2022DW-04-01).

### 2.3. DSS-Induced Colitis and Treatment

Mice were divided into the following six groups (*n* = 8) according to body weight: control, DSS, low-dose baicalin, medium-dose baicalin, high-dose baicalin, and 5-ASA as a positive control. Experimental colitis was induced by administering 3.0% DSS through the drinking supply for the first seven days, after which the drinking supply was replaced with distilled water. The following treatments were then administered for seven days via oral gavage: Control and DSS groups received distilled water; low-dose, medium-dose, and high-dose baicalin groups received 25, 50, and 100 mg/kg BW baicalin, respectively; and the 5-ASA group received 200 mg/kg BW 5-ASA. Throughout the experiment, mice body weight, stool consistency, and fecal blood were recorded every day [18]. The disease activity index (DAI) was scored according to the specific criteria as shown in Table 1 [19]. The DAI score was the mean of the total score of the three parts.

### 2.4. Hematoxylin and Eosin Staining

1 cm of tissue from the rectal end of the colon was harvested and fixed in 4% paraformaldehyde. After 24 hours, the tissue was rinsed and then dehydrated with increasing concentrations of ethanol, cleared in xylene, embedded in paraffin, and cut into 4–5 *μ*m thick tissue sections. Tissue sections were placed on glass slides and stained with H&E using standard procedures. The colon tissue's pathological changes were then observed using a light microscope [20].

### 2.5. RNA Analysis

Total RNA was extracted from mouse colon tissue using TRIzol reagent (Invitrogen). cDNA was generated using the HiScript II RT SuperMix for PCR (Vazyme). The mRNA level was quantified using ChamQ SYBR Green qPCR Master Mix (Vazyme) and determined by normalizing the expression of each target gene to that of *β*-actin using the 2^−△△t^ method. Detailed information of the primers used for RNA analysis is listed in Table 2.

### 2.6. Western Blotting

Proteins were extracted from colon tissue samples and separated by size using SDS-PAGE with 8%, 10%, or 12% gradient (Bis-Tris Midi Gel, Invitrogen) polyacrylamide gels, transferred to a blotting membrane, incubated with primary antibodies against caspase-1, ZO-1, MUC2, claudin-4, NLRP6, claudin-5, E-cadherin, and *β*-actin, and then incubated with HRP-labeled secondary antibodies. The blotting membrane was incubated with HRP substrate, and the immunoreactive bands were visualized using the ChemiDoc^TM^ XRS + system. *β*-Actin was used as a loading control to normalize the levels of detected protein on the blotting membrane.

### 2.7. Immunohistochemistry

Paraffin-embedded colon specimens of 4 *μ*m thickness were analyzed for MUC2, IL-18, and NLRP6 by immunohistochemistry. After antigen retrieval, samples were incubated with primary antibodies overnight at 4°C followed by incubation with biotin-labeled secondary antibodies and streptavidin-HRP for 30 minutes each at room temperature. Samples were then stained with 3-3-diaminobenzidine, followed by counterstaining with hematoxylin. Finally, specimens were dehydrated, cleared, and mounted on glass slides with coverslips. Immunoreactivity was observed using a light microscope.

### 2.8. ELISA

Mouse serum was used to detect TNF-*α*, IL-6, and IL-1*β* antibodies by ELISA (Multi Sciences) according to the manufacturer's instructions.

### 2.9. Alcian Blue and Periodic Acid-Schiff Staining

Paraffin-embedded colon specimens of 4 *μ*m thickness were analyzed for goblet cells by AB-PAS staining. Samples were stained with Alcian Blue staining solution, treated with 1% aqueous periodic acid, and stained with Schiff's reagent, and then, nuclei were lightly stained with hematoxylin. Samples were differentiated with acid alcohol, washed with Scott's tap water, and then finally dehydrated, cleared, and mounted on glass slides with coverslips. The number of goblet cells was determined by counting the Alcian Blue-positive vacuoles under a light microscope.

### 2.10. Statistical Analysis

GraphPad Prism (version 8.0.1; GraphPad Software, Inc.; San Diego, CA, USA) was used to analyze and construct the graphs in this study. Data were expressed as mean ± standard error of the mean (SEM). The Shapiro–Wilk test was used to assess the normality and homogeneity of the results. One-way analysis of variance (ANOVA) by Tukey's multiple comparisons test was also used to analyze the experimental results. Statistical significance was defined by *P* < 0.05.

## 3. Results

### 3.1. Baicalin Ameliorates DSS-Induced Colitis

Mice were given DSS through the drinking supply for seven days to establish the experimental colitis model (Figure 1(a)), which manifested as weight loss, diarrhea, and hematochezia. However, after the oral administration of baicalin at a series of doses and 5-ASA for another seven days, the weight loss associated with colitis was significantly reversed especially in the high-dose baicalin (100 mg/kg) group and the 5-ASA group (Figure 1(b)). The DAI score of the high-dose baicalin (100 mg/kg) group was lower than that of the DSS colitis model group, while the DAI score of the other four groups did not decrease compared with that of the DSS group (Figure 1(e)). Shortening of the colon is a typical symptom in colitis models (Figures 1(c) and 1(d)). As shown in Figures 1(b)–1(e), administration of baicalin (100 mg/kg) and 5-ASA could significantly reverse this symptom.

### 3.2. Baicalin Decreases Colon Inflammation in Colitis

Histological analysis of colon tissue in colitis mice often shows structural abnormalities, crypt deformation, and inflammatory cell infiltration. Mucosal damage was shown to be significantly improved after the administration of baicalin (100 mg/kg) and 5-ASA (Figures 2(a)–2(b)). In order to evaluate the anti-inflammatory effects of baicalin, mRNA and protein levels of proinflammatory cytokines, including IL-6, IL-1*β*, and TNF-*α*, were determined. Results show that mRNA expression and protein production of proinflammatory cytokines decreased after administration of baicalin in a dose-dependent manner. However, there was no difference between the DSS group and the 5-ASA group (Figures 2(c)–2(i)).

### 3.3. Baicalin Ameliorates Intestinal Barrier Damage

Disorder of the intestinal barrier is an important feature of colitis. An important part of the intestinal barrier is tight junctions (TJs), which are influenced by proteins such as ZO-1, E-cadherin, claudin-4, claudin-5, and claudin-2. The expression of TJs was assessed in mRNA and protein levels (Figures 3(a)–3(f)). Our study demonstrated that administration of baicalin could significantly upregulate both the mRNA expression and protein production of tight junction protein complexes in colon tissue.

### 3.4. Baicalin Protects Goblet Cells by Activating NLRP6 Inflammasomes

NLRP6 inflammasomes play a crucial role in the regulation of the mucosal barrier. DSS treatment resulted in colon tissue with downregulated mRNA expression levels of NLRP6 and apoptosis-associated speck-like protein containing a C-terminal caspase recruitment domain (ASC), while mRNA expression levels of caspase-1 were upregulated. Administration of baicalin reversed this dysregulated immune response in a dose-dependent manner, as shown by the upregulation of NLRP6 and ASC expression and the downregulation of caspase-1 expression (Figures 4(a)–4(d)). At the protein level, we found that baicalin could significantly increase the production of NLRP6 and decrease the production of caspase-1 (Figures 4(e)–4(g)). In order to visibly represent the expression of NLRP6 in colonic tissue, we did an immunohistochemistry analysis. As shown in Figures 4(h)–4(i), the distribution of NLRP6 protein was localized predominantly on the colon epithelial cell membrane in the DSS/baicalin (100 mg/kg) group and the DSS/5-ASA group. Also, we found that the administration of baicalin in a high dose could increase the level of IL-18 both in mRNA expression and in protein production (Figures 4(d) and 4(j)).

Another role of NLRP6 inflammasomes is to regulate goblet cells' mucus production, which may contribute to the formation of the mucosal layer. AB-PAS staining (Figures 5(a) and 5(b)) results showed that the administration of baicalin protected goblet cells, but not in a dose-dependent manner. Furthermore, we detected mRNA expression and protein production of mucins. As shown in Figures 5(d)–5(f), the protein levels of MUC2 were significantly downregulated in the DSS group but were upregulated after baicalin treatment and 5-ASA treatment. Altogether, this suggests that the activation of NLRP6 inflammasomes may be a potential mechanism by which baicalin protects goblet cells.

## 4. Discussion

UC is a major health problem that not only affects quality of life but also leads to a higher risk of colorectal cancer (CRC). Currently, biologic drugs for the treatment of UC are mainly targeted at mechanisms of immune dysregulation, such as TNF-*α* and IFN-*γ*. Intestinal barrier damage is a major characteristic of UC, and intestinal barrier dysfunction is the first and most important step of UC development [21]. Immune impairment and promotion of inflammatory responses caused by gut microbes and small molecules are further exacerbated when the gut barrier is compromised [22]. Inhibiting inflammation and rebuilding the intestinal barrier is a core strategy for UC treatment. According to UC management guidelines, the goal of UC treatment has been shifted from targeting immune dysregulation to the healing of the mucosa [4]. In the intestinal barrier, the two-layer mucosal barrier plays a crucial role in resisting injury from gut microbiota. Decreased goblet cell count and thinning of the mucus layer, with a lowered expression of MUC2, are commonly seen both in patients with UC and in animal models of colitis. Protecting goblet cells and rebuilding the mucosal barrier are a potential clinical treatment of UC. In this study, we demonstrated that baicalin has a protective effect on goblet cells and promotes the production of mucus in the large intestine.

NLRP6 inflammasomes are highly expressed in intestinal epithelial cells. They consist of an NLR sensor, an effector protein [23, 24]. NLRP6 inflammasomes have an important role in regulating intestinal epithelial cells by controlling the production of IL-18 and antimicrobial peptides to inhibit the expansion of gut microbiota [25], and coordinating goblet cell mucin granule exocytosis [26]. NLRP6-knockout mice appear to be more susceptible to DSS-induced colitis than wild-type (WT) mice, possibly due to defective autophagy and reduced mucus secretion in goblet cells [27]. Similar to previous studies [28], we found that decreastion of NLRP6 in the colonic tissue of colitis mice (Figures 4(e) and 4(h)). In addition, the production of IL-18, which promotes the secretion of mucus from goblet cells, was reduced (Figure 4(i)). Activation of NLRP6 is a potential strategy to deal with goblet cell and mucosal layer damage.

Fortunately, several studies have reported that natural flavonoids may protect mice from colitis by modulating an inflammasome-independent mechanism by which NLRP6 reprograms the gut microbiota [29]. Based on previous studies, baicalin, a type of flavonoid, is a potential new drug for colon diseases shown to have an excellent therapeutic effect on colitis and colitis-associated cancer [30]. In this study, DSS-induced colitis was used as the experimental model. The results showed that treatment with baicalin could reduce the symptoms of colitis as evidenced by the decrease in DAI scores, and the inhibition of weight loss and colon shortening (Figure 1). In addition, treatment with baicalin showed significant anti-inflammatory effects both in colon tissue and in serum (Figure 2). Specifically, treatment with baicalin decreased the serum level of IL-6 (Figure 2(g)), which is correlated with the clinical and histopathological severity of UC. Moreover, this study revealed that treatment with a high dose of baicalin had an excellent effect on activating NLRP6 inflammasomes (Figure 4), protecting goblet cells, and promoting mucus secretion (Figures 5 and 6).

## 5. Conclusion

Baicalin promotes the secretion of mucus by goblet cells through the activation of NLRP6 inflammasomes, thereby protecting mucosal barrier function.

## Figures and Tables

**Figure 1:** Baicalin attenuates DSS-induced colitis in mice. (a) Animal experiment design. (b) Body weight changes during the experiment. Representative colon length (c) and images of colons (d). (e) Evaluation of the disease activity index (DAI). Data are presented as mean ± SEM (*n* ≥ 5). ^*∗*^*P* < 0.05 vs. DSS group; ^*∗∗*^*P* < 0.01 vs. DSS group.

**Figure 2:** Baicalin inhibits inflammation of colon tissue. Representative images of H&E staining (a) and histological scores (b). Scale bar: 100 *μ*m. The mRNA expression levels of IL-1*β* (c), IL-6 (d), TNF-*α* (e), and IL-10 (f) in colon tissue. The protein levels of IL-6 (g), IL-1*β* (h), and TNF-*α* (i) in serum. Data are presented as mean ± SEM (*n* ≥ 5). ^*∗*^*P* < 0.05 vs. DSS group; ^*∗∗*^*P* < 0.01 vs. DSS group.

**Figure 3:** Baicalin regulates tight junctions of colon tissue. (a–e) The mRNA expression levels of ZO-1, E-cadherin, claudin-5, claudin-4, and claudin-2 in colon tissue. (f) The protein levels of ZO-1, E-cadherin, claudin-4, and claudin-5 in colon tissue determined by immunohistochemistry. Data are presented as mean ± SEM (*n* ≥ 5). ^*∗*^*P* < 0.05 vs. DSS group; ^*∗∗*^*P* < 0.01 vs. DSS group.

**Figure 4:** Baicalin activates NLRP6 inflammasomes. The mRNA expression levels of NLRP6 (a), ASC (b), caspase-1 (c), and IL-18 (d) in colon tissue. (e–g) The protein levels of NLRP6 and caspase-1 in colon tissue determined by Western blotting. (h, i) Representative images of immunohistochemical staining of NLRP6 and the quantification of NLRP6 by ImageJ. (j) Representative images of immunohistochemical staining of IL-18. Scale bar: 100 *μ*m. Data are presented as mean ± SEM (*n* ≥ 5). ^*∗*^*P* < 0.05 vs. DSS group; ^*∗∗*^*P* < 0.01 vs. DSS group.

**Figure 5:** Baicalin protects the intestinal mucosal barrier. (a, b) Representative images of AB/PAS staining and goblet cell count in each crypt. Scale bar: 100 *μ*m. (c–e) The mRNA expression and protein levels of MUC2 in colon tissue. (f, g) Representative images of immunohistochemical staining of MUC2 and the quantification of MUC2 by ImageJ. Scale bar: 100 *μ*m. Data are presented as mean ± SEM (*n* ≥ 5). ^*∗*^*P* < 0.05 vs. DSS group; ^*∗∗*^*P* < 0.01 vs. DSS group.

**Figure 6:** Mechanism diagram of baicalin protecting the intestinal mucosal barrier through activating NLRP6 inflammasomes.

**Table 1:** Disease activity index score.

Score	Weight loss (%)	Stool consistency	Gross bleeding
0	None	Normal	Negative
1	1–5	—	—
2	6–10	Loose stools	Hemoccult positive
3	11–15	—	
4	More than 15	Watery diarrhea	Bleeding

**Table 2:** qPCR primer sequences.

Gene	Primer	Sequence (5′-3′)
*β*-Actin	F	CTCATGAAGATCCTGACCGAG
	R	AGTCTAGAGCAACATAGCACAG

IL-6	F	CCACTTCACAAGTCGGAGGCTTA
	R	AGTGCATCATCGTTGTTCATAC

TNF-*α*	F	AAGGCCGGGGTGTCCTGGAG
	R	AGGCCAGGTGGGGACAGCTC

IL-1*β*	F	GAAATGCCACCTTTTGACAGTG
	R	TGGATGCTCTCATCAGGACAG

MUC2	F	TGTGTTTCAGGCTCCATCAC
	R	TGCAGCCATTGTAGGAAATC

NLRP6	F	TGGAGCCTCCTGCTCCAG
	R	GCGAGGCCACATCTCGAATA

Caspase-1	F	CCTGTCAGGGGCTCACTTTT
	R	GGTCACCCTATCAGCAGTGG

ASC	F	TGACAGTGCAACTGCGAGAA
	R	GTGAGCTCCAAGCCATACGA

IL-18	F	GGCTGCCATGTCAGAAGACT
	R	GTCTGGTCTGGGGTTCACTG

IL-10	F	CTTACTGACTGGCATGAGGATCA
	R	GCAGCTCTAGAGCATGTGG

Zo-1	F	GTCCCTGTGAGTCCTTCAGC
	R	TAGGGTCACAGTGTGGCAAG

E-cadherin	F	AACCCAAGCACGTATCAGGG
	R	ACTGCTGGTCAGGATCGTTG

Claudin-5	F	CCTTCCTGGACCACAACATC
	R	CGCCAGCACAGATTCATACA

Claudin-4	F	ACGTCATCCGCGACTTCTAC
	R	TTGTCGTTGCTACGAGGTGG

Claudin-2	F	CAAAGCCAAGAGTGAGTTCAA
	R	TCATTCTACCCTCAGCAGCA

## Data Availability

The data used to support the findings of this study are available from the corresponding author upon request.
